The article "Role of cytochrome P450 in drug interactions" was retracted in 2014. Reasons: plagiarism; overlap with other authors' work; no approval from an author; concerns about the authorship.

# Role of cytochrome P450 in drug interactions

**DOI:** 10.1186/1743-7075-5-27

**Published:** 2008-10-18

**Authors:** Zakia Bibi

**Affiliations:** 1 Department of Chemistry, University of Karachi, Karachi-75270, Pakistan

## Abstract

Drug-drug interactions have become an important issue in health care. It is now realized that many drug-drug interactions can be explained by alterations in the metabolic enzymes that are present in the liver and other extra-hepatic tissues. Many of the major pharmacokinetic interactions between drugs are due to hepatic cytochrome P450 (P450 or CYP) enzymes being affected by previous administration of other drugs. After coadministration, some drugs act as potent enzyme inducers, whereas others are inhibitors. However, reports of enzyme inhibition are very much more common. Understanding these mechanisms of enzyme inhibition or induction is extremely important in order to give appropriate multiple-drug therapies. In future, it may help to identify individuals at greatest risk of drug interactions and adverse events.

## Introduction

The cytochrome P450 (P450 or CYP) isoenzymes are a group of heme-containing enzymes embedded primarily in the lipid bilayer of the endoplasmic reticulum of hepatocytes, it takes part in the metabolism of many drugs, steroids and carcinogens [1]. The most intensively studied route of drug metabolism is the P450-catalysed mixed-function oxidation reaction which conforms to the following stoichiometry

NADPH + H^+ ^+ O_2 _+ RH → NADP^+ ^+ H_2_O + ROH

where, RH represents an oxidisable drug substrate and ROH is the hydroxylated metabolite, the overall reaction being catalysed by the enzyme P450. At the present time a number of CYP isoenzymes are expressed in each mammalian species including humans [2], many of these have specific role involving anabolic steroids and are localized in the liver. The present system of nomenclature for the various CYP isozymes employs a three-tiered classification based on the conventions of molecular biology: the family (members of the same family display > 40% homology in their amino acid sequences), subfamily (55% homology), and individual gene [3].

This pedigree is indicated by, respectively, an Arabic numeral (family), a capital letter (subfamily) and another Arabic numeral (gene), e.g. CYP1A2. The enzymes transforming drugs in humans belong to the CYP families 1–4 and more than 30 human CYP isozymes have been identified to date. It has been estimated that 90% of human drug oxidation can be attributed to six main enzymes (CYP1A2, 2C9, 2C19, 2D6, 2E1 and 3A4/5). The activities of the CYP2C19 [4-7] and CYP2D6 [8-14] enzymes are biomedically distributed in the population, allowing classification of individuals as either extensive (EM) or poor metabolizers (PM). The concept that most drug oxidations are catalysed primarily by a small number of P450 enzymes is important in that the approaches to identifying drug-drug interactions are feasible, both *in vivo *and *in vitro*.

More side-effects of drugs and drug-drug interactions are being reported, as highly effective drugs are developed and multiple-drug therapies are increasingly used. Drug interactions involving the P450 isoforms generally are of two types: enzyme induction or enzyme inhibition. Common substrates, inhibitors and inducers of P450 isozymes. Enzyme inhibition reduces metabolism, whereas induction can increase it. In general, high-extraction drugs are less affected by these interactions than low-extraction drugs. As have been shown in recent deaths [15,16] caused by dysrhythmia or bone marrow (haematopoietic) inhibition due to combined administration of terfenadine and ketoconazole [17,18], erythromycin [19] and itraconazole [20], and sorivudine and fluoropyrimidines, are clinically important and severe interactions do occur. Furthermore, side-effects due to drug-drug interactions in elderly patients because of their reduced physiological functions are reportedly becoming more frequent and associated with more severe symptoms; thus, much importance is being attached to information about drug-drug interactions when giving any drug therapy. A number of reviews of these interactions have been published [21-63].

In recent years, access to human tissue samples was not possible in Japan. However, characterization of P450 reactions catalysed by human P450s have been carried out in the United States and Europe. The availability of the recombinant human P450s expressed in various systems has also facilitated studies of their catalytic selectivity [64]. Thus, it is now relatively straightforward to determine *in vitro *interactions in which P450s oxidizes a particular drug and which drugs can inhibit oxidations catalysed by this P450. Thus, it is possible to perform logical *in vivo *studies to test the relevance of *in vitro *findings [65,66]. This review discusses interactions and their clinical management.

### P450 enzyme classification

In man there are around 30 CYP enzymes which are responsible for drug metabolism and these belong to families 1–4. It has been estimated, however, that 90% of drug oxidation can be attributed to six main enzymes: CYP 1A2, 2C9, 2C19, 2D6, 2E1 and 3A4 [6]. The most significant CYP isoenzymes in terms of quantity are CYP3A4 and CYP2D6. CYP3A4 is found not only in the liver but also in the gut wall, where it may serve as a primary defence mechanism. The bulk of drugs acting on the CNS (Central Nervous System), with the exception of volatile anaesthetic agents, are metabolized by this enzyme.

### CYP1A subfamily

#### CYP1A1 and CYP1A2

The CYP1A family consists of two enzymes, 1A1 and 1A2. CYP1A1 is not significantly expressed in the liver. It is found mainly in the lungs, mammary glands, placenta and lymphocytes. It is an enzyme involved in the inactivation of procarcinogens and is highly induced by polycyclic aromatic hydrocarbons (PAHs), which are found in cigarette smoke [7]. There is a strong association between the activity of CYP1A1 and the risk of lung cancer [8]. CYP1A2 is expressed mainly in the liver and is induced by cigarette smoking [9]. It is also induced by the ingestion of some foodstuffs such as cruciferous vegetables as well as barbecued or charbroiled food [10]. Some drugs such as omeprazole may induce CYP1A2 activity [11]. Drugs which are known to be metabolized by CYP1A2 include theophylline, caffeine, imipramine, paracetamol and phenacitin [12]. Alteration in CYP1A2 activity, for example by smoking, may alter the requirements for theophylline among asthmatics [13] and haloperidol among psychiatric patients [14]. Caffeine metabolism is also induced by smoking and explains the increased tolerance to caffeine among smokers [15].

#### CYP2 family

CYP2A6, previously known as coumarin hydroxylase, is a relatively unimportant enzyme in terms of the number of substrates which it metabolizes, one of the substrates broken down by this enzyme is nicotine. Differences, both racial and inter individual, in expression levels are thought to be related to the propensity to develop nicotine dependence [16].

*CYP2C subfamily*: is one of the most important families and consists primarily of two enzymes, *CYP2C9 and CYP2C19*.

*CYP2C9*: Among the substrates of CYP2C9 is the anticoagulant warfarin, which exists in two distinct isoforms of which the S-form is the most important and this is metabolized by CYP2C9 [17]. There are a number of polymorphisms of the gene that encode this enzyme resulting in *poor metabolic *status. These patients may be difficult to stabilize on standard warfarin regimens [18]. Other drugs metabolized by CYP2C9 include non-steroidal anti-inflammatory drugs (NSAIDs) (including COX-2 selective inhibitors), the hypoglycemic agent tolbutamide, phenytoin and the angiotensin-II receptor antagonist losartan.

*CYP2C19 *has a number of commonly used substrates including the benzodiazepine diazepam, the proton pump inhibitor omeprazole, propanolol and the antidepressive amitriptyline [19]. A number of important abnormal variants of this enzyme exist, one of these has important clinical consequences. It has been demonstrated that poor metabolizers who are prescribed proton-pump inhibitor omeprazole as part of therapy against *Helicobacter pylori *infection may have significantly better clinical outcomes as compared to a group of patients homozygous for the normal, i.e. wild-type, alleles [20].

#### CYP2D subfamily

*CYP2D6*. A large number of drugs are metabolized by this enzyme including a number of anti-arrhythmics such as flecanide and encainide, tricyclic antidepressants, some beta-blockers and a number of selective serotonin re-uptake inhibitors. It is of particular relevance to anesthetics because a number of commonly used analgesics, including codeine and tramadol, are broken down by this enzyme [21]. Previously named debrisoquine hydroxylase [22], was one of the first to be categorised following recognition that the metabolism of the hypotensive agent debrisoquine was abnormal in a proportion of individuals. It was renamed CYP2D6 after the parent gene was cloned and the enzyme categorized [23]. To date, more than 70 polymorphisms of CYP2D6 have been catalogued. The majority of these enzymes result in a poor metaboliser phenotype as opposed to the normal, i.e. extensive metabolize phenotype. In addition, a number of genotypes exist where gene duplication results in an ultra rapid metabolize status. These patients eliminate CYP2D6 substrates faster than normal and in case of pro-drugs such as codeine are at greater risk of opiate related side-effects [24].

#### CYP2E1

The CYP2E family contains only one enzyme, CYP2E1 (previously dimethylnitrosamine N-demethylase), which is responsible for the metabolism of small organic compounds such as alcohol and carbon tetrachloride as well as the halogenated anaesthetic agents halothane, enflurane, diethyl ether, trichloroethylene, chloroform, isoflurane and methoxyflurane [25]. It is also responsible for the breakdown of many low molecular weight toxins and carcinogens, many of which are used in manufacturing and dry cleaning industry, including benzene, styrene, acetone, vinyl chloride and N-nitrosamines. Some of these substances are pro carcinogens which are activated by CYP2E1. There are gender differences in the expression of the enzyme, obesity and fasting may also affect its activity [26]. This may provide a putative explanation for obesity related cancers [27].

Because of the key role of CYP2E1 in the biodegradation of a number of environmental carcinogens, the enzyme has been studied closely in relation to the causation of neoplasia. For example, in China an association was detected between polymorphisms of CYP2E1 and oesophageal and gastric cancer [28]. There is also mounting evidence that CYP2E1 may be a key factor in the pathogenesis of alcoholic liver disease [29]. The exact role of CYP2E1 is unclear, although the enzyme is induced by both alcohol and nicotine [30], and may explain the higher ethanol elimination rates among smokers [31].

#### CYP3A subfamily

*CYP3A4 *is the most abundantly expressed drug metabolizing enzyme in man responsible for the breakdown of over 120 different medications and is thus an important area for study with respect to enzyme based drug interactions. Among the drugs metabolized are sedatives such as midazolam, triazolam and diazepam, the antidepressives amitriptyline and imipramine, the anti-arryhthmics amiodarone, quinidine, propafenone and disopyramide, the antihistamines terfenadine, astemizole and loratidine, calcium channel antagonists such as diltiazem and nifedipine and various antimicrobials and protease inhibitors [6].

#### Mechanism of pharmacokinetic drug-drug interaction

##### Inhibition

Inhibition is reduced enzyme activity due to direct interaction with a drug. This process usually begins with the first dose of the inhibitor, and the start and finish of inhibition correlate with the half-lives of the drugs involved [67]. There are three basic types of enzyme inhibition (competitive, non-competitive and uncompetitive), and clinical effects are influenced by these basic mechanisms [68,69].

The first type is competitive inhibition between inhibitor and substrate for the same binding site on an enzyme. The size and flexibility of the binding site of the microsomal P450 with which we are concerned here are unknown. For example, when single oral doses of metoprolol (50 mg), a beta-adrenoceptor blocking agent and/or propafenone (150 mg) were administered, or when the two drugs were given in combination to healthy subjects, an approximately two-fold reduction in the oral clearance of etoprolol was observed when propafenone was included. The dose of metoprolol should be reduced when propafenone is also given [70]. Similar drug-drug interactions are seen in the combined administration of thioridazine and propranolol (CYP2D6) [71], fluoxetine and desipramine (CYP2D6) [72], omeprazole and diazepam (CYP2C19) [73-75], tolbutamide and phenytoin (CYP2C9) [32], and diltiazem and cyclosporin (CYP3A) [76-78].

The most typical example of the second type of drug-drug interaction includes that of terfenadine and erythromycin [19]. The combined use of these drug, terfenadine, and macrolides (antibiotics) or ketoconazole prolongs electrocardiographic QT intervals, thereby triggering a specific cardiac dysrhythmia known as torsades de pointes' [18]. The mechanism of this interaction is considered to occur when a nitro compound, namely a metabolite demethylated by P450, forms a complex with P450. Since macrolides are catalysed by CYP3A, metabolites selectively form CYP3A and a stable enzyme-substrate complex [34,79-81].

In consequence, it has been reported that the metabolism of drugs like carbamazepine [81-83], midazolam [84-86] and cyclosporin [87] are catalysed by CYP3A, and their plasma concentrations are increased when its metabolism is inhibited by combined use with erythromycin. A P450 species that catalyzes the metabolism of terfenadine was identified recently as CYP3A [88,89] during investigations of the mechanism of interactions with macrolides.

Another type is non-competitive inhibition, where the inhibitor binds at a site on the enzyme distinct from the substrate, as happens in classical studies of enzymology. Such examples include interactions between cimetidine and a number of drugs. The duration of this type of inhibition may be longer if new enzymes are synthesized after the inhibitor drug is discontinued. Cimetidine is bound to P450 and produces a stable cytochrome-substrate complex. It is the formation of this complex which prevents access of other drugs to the P450 system. Cimetidine does not inhibit conjugation mechanisms including glucuronidation, sulphation and acetylation, or deacetylation or ethanol dehydrogenation. It binds to the haem portion of P450 and is, thus, an inhibitor of phase I drug metabolism reactions (i.e. hydroxylation, dealkylation) [90-92]. Although generally recognized as a nonspecific inhibitor of this type of metabolism, cimetidine does demonstrate some degree of specificity. Since every molecular species of P450 has a haem portion, it is possible for cimetidine to nonspecifically inhibit any drug that is metabolized by any molecular species. However, in a recent study that compared the inhibitory effect of several P450 isozymes in a study using drugs such as ketoconazole, clotrimazole, miconazole, fluconazole, secnidazole and metronidazole, all imidazole derivatives [92,93], it was reported that isoniazid, an antituberculous drug, inhibits the metabolism of phenytoin [94]. As for its inhibitory mechanism, it is conceivable that there is an interaction between the hydrazino group of isoniazid and the haem portion of P450. As far as ethinylestradiol, an oral contraceptive, is concerned, the CYP3A isozyme is one of the major forms involved in its 2-hydroxylation [93,95,96]. Guengerich reported that *in vitro *it is a relatively effective and selective mechanism-based inactivator of CYP3A4 [96]. This inactivation is due in part to the presence of an ethynyl moiety, which is also found in many inactivators [93-97].

##### Induction

The effect of induction is simply to increase the amount of P450 present and speed up the oxidation and clearance of a drug [67]. It is rather difficult to predict the time-course of enzyme induction because of several factors, including the drug half-life and enzyme turnover, which determine the time-course of induction. A complicating factor is that the time-course of induction depends on the time required for enzyme degradation and new enzyme production. The short half-life of rifampicin results in enzyme induction (CYP3A4, CYP2C), apparent within 24 h, whereas phenobarbital, which has a half-life of 3–5 days, requires ≅1 week for induction (CYP3A4, CYP1A2, CYP2C) to become apparent. These enzyme-induction reactions also occur with smoking and long-term alcohol or drug consumption and can reduce the duration of action of a drug by increasing its metabolic elimination. Of all these drugs, the clinically most problematic drug involves the rifampicin series [98-106] which includes antiepileptic drugs such as phenobarbital [107,108], carbamazepine [109,110] and phenytoin [108,110] and antituberculous drugs [110]. The CYP1A2 enzyme can be induced by exposure to polycyclic aromatic hydrocarbons, such as are found in char-grilled foods and cigarette smoke [111,112]. Most human CYP2C and 3A subfamily proteins are induced by barbiturates [113], while human CYP2E1 is inducible by ethanol and isoniazid, although the mechanism involved is complex [114,115]. One example has been described by Lee *et al*. [99] who reported that changes in the pharmacokinetics of prednisolone were caused by administration or discontinuation of rifampicin. Pharmacokinetic studies of prednisolone (1 mg/kg) in patients over a 1-month period of rifampicin co-treatment or after its withdrawal revealed significant changes in the area under the curve (AUC), total body clearance, non-renal clearance and half-life. As mentioned earlier, rifampicin is possibly associated with plural molecular species of P450 (several isozymes), but mainly, a large increase in the CYP3A content often becomes a problem, while phenobarbital, carbamazepine and phenytoin, antiepileptic drugs, also induce CYP3A [32]. Thus, appropriate therapeutic effects can hardly be obtained unless the doses are increased significantly, since plasma concentrations are not elevated in patients receiving these drugs which are metabolized by CYP3A. The P450 isoenzymes induced by exposure to polycyclic aromatic hydrocarbons, such as those found in char-grilled foods and cigarette smoke, are CYPlAl and CYP1A2 [116,117]. CYPIA2 is a molecular species of P450 which participates in the metabolism of several important drugs such as theophylline and propranolol and, since its activity is enhanced by smoking and eating grilled meat or cruciferous vegetables, it is difficult to obtain therapeutic effects. Although CYP2C9, CYP2C19 and CYP2E1 are also induced, no specific inducers of CYP2D6 have yet been identified clearly. However, it appears to be inducible.

#### Mechanism of non-microsomal pharmacokinetic drug-drug interactions

Sixteen Japanese patients died when given both sorivudine and fluoropyrimidines orally. Sorivudine is a potent inhibitor of hepatic dihydropyrimidine dehydrogenase, the enzyme responsible for the catabolism of fluoropyrimidines. Therefore, the fluoropyrimidine levels in these patients reached toxic levels due to the inhibition of dihydropyrimidine dehydrogenase by sorivudine [15,16].

### Clinical example of P450-based interactions

#### Terfenadine

Terfenadine is the first non-sedating H_1_-antihistamine drug. It is rapidly oxidized by CYP3A4 to two metabolites, acyclinol and an alcohol derived from the oxidation of a t-butyl methyl group [118]. The alcohol is further oxidized to a carboxylic acid by either CYP3A4 or dehydrogenase [119]. This carboxylic acid then binds to the H_1 _histamine receptor and should relieve allergy symptoms. The oxidation of terfenadine by CYP3A4 can be inhibited strongly by azole antifungal or antimicrobial agents such as ketoconazole [17,18] and erythromycin [19]. For example, Honing *et al*. [18] performed experiments on six healthy volunteers (four men and two women, aged 24–35 years). After achieving a steady-state while taking terfenadine (60 mg every 12 h for 7 days), daily concomitant oral ketoconazole (200 mg every 12 h) was added to the regimen. Pharmacokinetic profiles were obtained while subjects were taking terfenadine alone and after the addition of ketoconazole. Electrocardiograms were obtained at baseline, after 1 week of taking terfenadine alone, and at the time of the second pharmacokinetic profile after the addition of ketoconazole to the regimen. Serum concentrations of terfenadine and its acid metabolite and corrected QT intervals were obtained. All subjects had detectable levels of unmetabolized terfenadine after the addition of ketoconazole, associated with QT prolongation. Only two of the six subjects were able to complete the entire course of ketoconazole coadministration. Four subjects received a shortened period of ketoconazole therapy because of significant electrocardiographic repolarization abnormalities. There was a significant reduction in the AUC of the acid metabolite of terfenadine during ketoconazole administration. Therefore, the blood concentration of terfenadine increased. High blood levels of terfenadine have been associated with cardiac problems including dysrhythmias, torsade de pointes, and abnormal ventricular rhythms. For this reason, very carefully controlled co-administration of terfenadine is advised.

#### Cimetidine

Cimetidine inhibits antihistamine H_2_-receptor binding and is used in the treatment of gastric ulcers. The mechanism of inhibition appears to involve the imidazole ring of cimetidine with competitive binding, which is not present in ranitidine [90,91]; it also exhibits selective inhibition of reactions catalysed by CYP2D6 and 3A4 [90,92-120]. For example, unlike ranitidine, cimetidine significantly increased the maximum plasma concentration (C_max_), AUC and the total amount of disopyramide excreted unchanged in the urine, but the serum profile of mono-N-dealkyldisopyramide, a metabolite of disopyramide, was not affected significantly. Ranitidine had no significant effect on the pharmacokinetics of disopyramide and mono-N-dealkyldisopyramide. These results indicate that cimetidine, but not ranitidine, significantly increases the absorption of oral disopyramide [121]. Tanaka and Nakamura also investigated the effects of H_2_-receptor antagonists (cimetidine, ranitidine, and famotidine) on ethanol metabolism. In both aldehyde dehydrogenase (ALDH)-1 deficient subjects and in those with normal ALDH-1, the three H_2_-receptor antagonists and placebo had similar effects on the pharmacokinetic parameters of ethanol, i.e. peak time (t_max_), metabolic rate, C_max_, volume of distribution (Vd) and AUC. The AUC of acetaldehyde was slightly (*P *< 0.05) but significantly greater only after treatment with cimetidine; the C_max _and t_max _of acetaldehyde were unchanged [122]. As mentioned above, there are a number of drugs whose metabolism is inhibited when cimetidine is administered in combination [90-92].

#### Grapefruit juice

The opportunity for a food-drug interaction is an everyday occurrence, which can be particularly important when total drug absorption is altered. Recently, a chance observation led to the finding that grapefruit juice could markedly increase the oral bioavailability of a number of medications [123]. This article retraces discovery of this novel interaction and reviews the mechanism of action, summaries studied and predicted medications for an interaction, discusses possible active ingredient in the juice and considers clinical implications. In 1989 it was reported that coadministration of grapefruit juice with the calcium channel antagonist felodipine resulted in a large increase in serum felodipine concentrations, as well as an enhancement of the pharmacodynamic effects of the drug [124].

Some drugs exhibit a significantly increased (up to three-fold) mean oral bioavailability when co-administered with grapefruit juice. Bailey *et al *[125] reported that the inhibitory effect of grapefruit juice was discovered rather serendipitously in an interaction study with ethanol and felodipine, a 1,4-dihydropyridine calcium entry blocker. Flavonoids (e.g. quercetin, naringenin, kaempferol) found in large amounts in oranges, grapefruit and their juices are known to alter the activity of P450 enzymes (P450 isoenzyme). The mechanism of inhibition of drug oxidation probably involves intestinal CYP3A4. The major grapefruit-specific flavonoid is naringin, which can account for up to 10% of the dry weight. It is believed that this naringin mainly inhibits the enzyme (CYP3A) that metabolizes calcium antagonists. For example, interactions between benzodiazepines (e.g. midazolam, triazolam), antihistamines (e.g. terfenadine), immuno-suppressive drugs (e.g. cyclosporin) and grapefruit juice have been reported [125]. For example, Hukkinen *et al*. [126] studied 10 healthy young subjects who received a single 0.25 mg dose of triazolam with either 250 ml grapefruit juice or water. The plasma concentrations and effects of triazolam were measured up to 17 h. Grapefruit juice increased the AUC of triazolam in each subject and the C_max _in nine out of 10 subjects. The mean AUC of triazolam increased 1.5-fold (*P *< 0.001) and the peak concentration increased 1.3-fold (*P *< 0.05) following grapefruit juice. Grapefruit juice also postponed the peak time of triazolam from 1.6 to 2.5 h (*P *< 0.05). Grapefruit juice also increased the effects of triazolam, drowsiness being significantly (*P *< 0.05) enhanced. However, as it has been described in a paper [127] that other flavonoids (quercetin for example) may be major inhibitors of metabolism, the results of future studies are awaited with interest. On the other hand, it is reported that naringin also inhibits the demethylation (N-demethylation) of caffeine, metabolized by CYPIA2 [125]. It has already been established that, grape fruit juice is well known as potent inhibitors of cytochrome P450 3A4 activity. It increases bioavailability of several drugs known to be metabolized by CYP3A4, while on the other hand interact and block the activity of ciprofloxacin, ofloxacin, cefazolin and ceftizixime. Owing to clinical relevance of grapefruit juice-drug interactions, an investigation of drug interactions of two quinolones, ciprofloxacin and ofloxacin were investigated *in vitro *with all the fruit juices available locally at human body temperature [128]. A single glass of grapefruit juice has the potential to augment the oral bioavailability and to enhance the beneficial or adverse effects of a broad range of medications, even by juice consumed hours beforehand. Grapefruit juice acts by inhibiting presystemic drug metabolism mediated by CYP3A isoforms in the small bowel. The interaction appears particularly relevant for medications with at least a doubling of plasma drug concentration or with a steep concentration-response relationship or a narrow therapeutic index. Patients that appear particularly susceptible have high small bowel CYP3A4 content, hepatic insufficiency or a pre-existing medical condition, which predisposes to enhanced, excessive or abnormal drug effects [129].

#### Omeprazole

Omeprazole is a proton-pump inhibitor used widely for the treatment of gastric ulcers [53,62]. Omeprazole is converted to hydroxyomeprazole and omeprazole sulphone primarily by CYP2C19 and CYP3A4, respectively. Gugler and Jensen first reported that omeprazole reduced the plasma clearance and prolonged the half-life of phenytoin and diazepam but did not affect the apparent volume of distribution and plasma protein binding of either diazepam or phenytoin [130]. Recently, in a pharmacogenetic study, Anderson *et al*. [131] studied the effect of omeprazole treatment on diazepam plasma levels in 6 EM and 4 PM of omeprazole. Single i.v. doses of diazepam (0.1 mg/kg) were administered after 1 week of oral omeprazole (20 mg) and placebo. The slow metabolizers of omeprazole also metabolized diazepam slowly, exhibiting only half the diazepam plasma clearance of the others. The mean clearance of diazepam fell 26% after omeprazole in the rapid metabolizers, whereas the slow group showed no apparent interaction. Desmethyldiazepam was formed more rapidly in the rapid compared with the slow metabolizers, which is a logical consequence of the rate of diazepam metabolism. In the light of these results, omeprazole appears to be a competitive inhibitor of CYP2C19, and involved in its metabolism. These data show that omeprazole interferes with the elimination of other drugs by inhibiting the mixed function oxidases of human liver. Other acid pump inhibitors (lansoprazole or pantoprazole) are also mainly metabolized by CYP2C19. For drugs metabolized by CYP2C19, such as 5-mephenytoin, imipramine or diazepam, their metabolism is inhibited [132].

#### Erythromycin

Erythromycin, an antimicrobial agent, is known to inhibit a number of drug oxidation reactions catalysed by CYP3A4 [80]. It inhibits the oxidation of terfenadine [19,133], cyclosporin [134] and numerous other drugs both *in vivo *and *in vitro *and erythromycin N-demethylation itself is catalysed by CYP3A4/5 [135,136]. However, not all CYP3A4 reactions are inhibited by erythromycin. As far as the above results are concerned, Guengerich [56] has made the following two proposals: i lack of inhibition of a reaction by erythromycin may not always be a reliable indication that the reaction is not catalysed by CYP3A4 and (ii) not all CYP3A4-catalysed reactions may be prone to erythromycin interactions. The reasons for this are not clear at the moment.

#### Cyclosporin

Cyclosporin is the most popular immunosupressant used in organ transplantation. The major pathway of cyclosporin metabolism is via CYP3A4 [137,138], with three major metabolites being formed [139]. Since cyclosporin is mainly used as an immunosuppressant for organ transplantation, the CYP3A4 level in the donor's liver as well as the recipient's liver, small intestine and other tissues must always be taken into consideration. For example, Lucey *et al*. [140] reported that a 40-year-old male liver allograft recipient had neurological dysfunction and renal failure while his cyclosporin blood levels were in the therapeutic range. CYP3A activity, using the [^14^C] erythromycin breath test, was reduced compared with that in controls, including other liver transplant recipients. Pretreatment with rifampicin, an inducer of CYP3A, increased enzyme activity. After treatment with rifampicin the patient was able to be rechallenged with cyclosporin at a dose almost twice that which had previously been toxic. The patient died during a second transplantation and the microsomal CYP3A content was found to be low in the first transplant liver. Lower blood levels of cyclosporin may have been achieved when the drug used for enzyme induction (rifampicin) has been given to the transplant patient for a long period [140].

#### Rifampicin

Rifampicin [98-106,141,142] and isoniazid [101] are key drugs used in the treatment of tuberculosis, while rifampicin is highly effective in inducing hepatic, drug metabolic P450 enzyme. When enzyme induction is achieved, the pharmacological effects of a specific drug may be reduced, since not only the metabolism of rifampicin itself, but also the metabolism of the other drug is accelerated [136]. The problem arises when doses are increased to reduce the effects of the combined drugs: increased serum concentrations of the combined drugs may possibly produce side-effects because of the lost enzyme induction if rifampicin is discontinued. Rifampicin is also known to induce CYP3A4 and CYP2C9 (e.g. cyclosporin, diazepam and steroids). As for dihydropyridine calcium channel blockers, it is quite possible that interactions with rifampicin may develop, since most of these drugs are metabolized by CYP3A4 [143-150,129].

## Conclusion

There are two main types of drug interaction: pharmacokinetic and pharmacodynamic. Pharmacokinetic interactions involve the effect of one drug on the absorption, metabolism, excretion or protein binding of another drug. On the other hand, pharmacodynamic interactions are caused by several effects (additive, synergistic or antagonistic effects) of the combined treatment at the site of biological activity, changing the pharmacological action of the drugs, even at standard blood concentrations. Pharmacokinetic interactions focused on P450 are described in this paper. The incidence of side-effects is markedly higher in the elderly and those with more severe symptoms. Thus, understanding the mechanism underlying drug interactions is useful, not only in preventing drug toxicity or adverse effects, but also in devising safer therapies for disease.

## Competing interests

The author declares that he has no competing interests.
